The article "A Novel Prognostic Stratified System Based on Tumor Budding and the Cell Nest Size in Ureter Urothelial Carcinoma" was retracted in 2023. Reasons: signs of a paper mill; suspected computer-generated content; unreliable results or conclusions; concerns about the data.

# A Novel Prognostic Stratified System Based on Tumor Budding and the Cell Nest Size in Ureter Urothelial Carcinoma

**DOI:** 10.1155/2022/6988237

**Published:** 2022-05-06

**Authors:** Jialin Li, Xinyue Li, Jing Yang

**Affiliations:** Department of Pathology, Jinzhou Medical University, Jinzhou, Liaoning, 40 Songpo Road, Linghe District, Jinzhou, Liaoning, China

## Abstract

At present, malignant tumor stratification based on the TNM stage is very important for predicting patient prognosis and selecting appropriate treatment. The prognostic factor of ureter urothelial carcinoma is mainly based on the stage according to AJCC (8th) TNM classification. None of the histomorphologic features is recommended to assess patient's prognosis. Recently, a novel three-tiered grading system based on tumor budding and the cell nest size (referred as TBNS system) has been applied to be highly prognostic for some squamous cell carcinomas, including esophageal, pulmonary, uterine cervix cancer, and endocervical endocarcinoma. In this study, we explored the application of this TBNS grading system in ureter urothelial carcinoma consisting 87 surgically resected cases and no neoadjuvant therapy. Tumor budding and the cell nest size were assessed and correlated with clinicopathological data and survival. The results showed that higher tumor budding, cell nest size, and TBNS grading system were strongly related to shorter overall survival (OS), disease-specific survival (DSS), and disease-free survival (DFS). Multivariate survival analysis showed the TBNS grading system to be closely related to the independent prognosis of DFS and DSS. In conclusion, the TBNS grading system based on tumor budding and cell nest size, if further validated, could satisfactorily predict the prognosis of uterine urothelial carcinoma and be applicable in routine pathologic description of this cancer type.

## 1. Introduction

Primary ureteral carcinoma is a rare tumor of the urinary system, which accounts for 5–10% of all urothelial carcinomas [1]. The incidence rate has increased significantly in recent years. The diagnosis of ureter carcinoma is difficult because the ureter is located behind the peritoneum, its position is concealed, and its anatomy is complex [2]. The tumor is prone to invasion and metastasis, and prognosis is poor. At present, the pTNM staging system developed by AJCC is recognized as the gold standard for reflecting the biological behavior and patient prognosis and guiding clinical treatment of ureteral cancer. However, even for patients with the same stage, the clinical outcomes of patients with the same surgical treatment and supplemented with radiotherapy and chemotherapy are different [3]. Therefore, it is an objective requirement of individualized therapy and precision medicine to find some morphological markers that can better reflect the biological behavior and prognosis of ureteral cancer and combine them with AJCC staging.

The article "A Novel Prognostic Stratified System Based on Tumor Budding and the Cell Nest Size in Ureter Urothelial Carcinoma" was retracted in 2023. Reasons: signs of a paper mill; suspected computer-generated content; unreliable results or conclusions; concerns about the data.

Tumor budding is a special histological morphology first described by Ueno et al. in colorectal cancer [4, 5] and has been described in many tumors [6–10]. According to the International Tumor Budding Consensus Conference criteria [11], tumor budding appears as a cluster of less than four tumor cells or a single tumor cell into the peritumoral stroma, which has high invasiveness, mobility, and epithelial-mesenchymal transition [12–14]. Emerging data demonstrate that tumor budding can predict poor prognosis in endometrial carcinoma [15], tongue carcinoma [16], pancreatic ductal adenocarcinoma [17], lung cancer [18], and uterine cervix [19]. The tumor cell nest size, defined as the smallest invasive tumor cluster within the entire tumor area, also relates to poor prognosis of the lung [20] and esophageal carcinoma [21] and so on. Recently, a novel three-tiered grading system combing the tumor budding activity and cell nest size, which is also referred as the TBNS (tumor budding/nest size) grading system, has been established for its high prognostic value in squamous cell carcinomas (SCCs) of various sites, including lung [20], oral cavity [22], esophagus [21], and larynx and hypopharynx [23]. Jesinghaus et al. [21] reported tumor budding and the cell nest size as strong prognostic predictors in esophageal carcinoma. Zare et al. [19] independently validated this grading system's application in uterine cervix carcinoma. Shi et al. [24] verified that the three-tiered grading system could be a perfect prognostic predictor which was superior to the FIGO grading and Silva pattern in endocervical adenocarcinoma.

These data showed the usefulness of the TBNS grading system for prognostic stratification in malignant tumors. However, the prognostic value of this novel grading system has not been investigated in ureter urothelial carcinoma yet. In the present study, we explored the prognostic ability of the TBNS grading system in ureter urothelial carcinoma.

## 2. Patients and Methods

### 2.1. Study Sample

We used 87 formalin-fixed paraffin-embedded (FFPE) tissue samples resected from ureter urothelial carcinoma patients between 2012 and 2017, collected retrospectively from the department of pathology, The First Affiliated Hospital, Jinzhou Medical University, China. The inclusion criteria were as follows: (1) all cases were pathologically diagnosed as ureteral urothelial carcinoma, (2) none of the patients received preoperative radiotherapy or chemotherapy, and (3) there is complete clinical data. Exclusion criteria are as follows: (1) complicating bladder cancer, (2) previous history of bladder cancer, (3) other tumors in the past, and (4) incomplete clinical data.

The article "A Novel Prognostic Stratified System Based on Tumor Budding and the Cell Nest Size in Ureter Urothelial Carcinoma" was retracted in 2023. Reasons: signs of a paper mill; suspected computer-generated content; unreliable results or conclusions; concerns about the data.

Tumor stage was reassessed according to the AJCC Cancer Staging Manual (8th) [3]. All patients underwent nephrectomy and full-length ureterectomy.

All patients were followed up by telephone from the first day after surgery, once every 3 months for 2 years and once every 6 months after 2 years. Patients who were lost to follow-up or in which tumor did not progress during follow-up were treated as the end point. Patients' informed consent was not required due to the retrospective nature of the study. This study was approved by the Institutional Review Board of The First Affiliated Hospital, Jinzhou Medical University (no. 202046). This study has been carried out in accordance with The Code of Ethics of the World Medical Association (Declaration of Helsinki) for experiments involving humans.

### 2.2. Histological Assessment

Two pathologists (Jing Yang and Jialin Li), blinded for clinicopathologic and clinical information, assessed the hematoxylin- and eosin-stained ureter urothelial carcinoma slides. When there was inconsistency in the assessment, the analysis was performed simultaneously under a multihead microscope to achieve unity. Urothelial carcinoma was divided into low and high grades according to the AJCC Cancer Staging Manual (8th) [3].

The assessment of morphology and score was according to the criteria in Jesinghaus et al. [21] and the three-tiered grading system criteria [19]. The tumor budding was defined as a single tumor cell or a group of ≤4 tumor cells present at the infiltrating edge of the malignant tumor and divided into three groups: without (1 point), low (2 point), and high budding (3 point) activity. Low and high budding activities were indicated by 1–14 and ≥15 buddings in 10 high-power fields (HPFs) (Figures 1(a) and 1(b)). If it is difficult to identify tumor budding, CK immunohistochemical staining can be used to assist in judgment.

The cell nest size was defined as a minimal size of invasive tumor cell nests and divided into four groups: large (>15 cells, 1 point), medium (5–15 cells, 2 points), small cell nests (2–4 cells, 3 points), and single-cell invasion (4 points) (Figure 1(c)). Then, the total scores were derived by adding tumor budding activity (1–3 points) and cell nest size (1–4 points) scores. This grading system was categorized as G1 (well differentiated, score 2 or 3), G2 (moderately differentiated, score 4 or 5), and G3 (poorly differentiated, score 6 or 7).

The article "A Novel Prognostic Stratified System Based on Tumor Budding and the Cell Nest Size in Ureter Urothelial Carcinoma" was retracted in 2023. Reasons: signs of a paper mill; suspected computer-generated content; unreliable results or conclusions; concerns about the data.

### 2.3. Immunohistochemical Staining

Paraffin sections of 4 *μ*m thickness were dewaxed and hydrated and repaired by citric acid antigen for 4 min. An endogenous peroxidase blocker was added for 10 min at room temperature. Add CK (mouse anti-human polyclonal antibody, Fujian Maixin Biotechnology Development Co. Ltd.) at 37°C for 60 min; add an appropriate amount of enzyme-labeled goat anti-rabbit lgG polymer at 37° for 20 min; DAB was added and placed at room temperature for 8 minutes. Rinse with running water and add hematoxylin staining solution for 40 seconds; then, put in hydrochloric acid alcohol, tap water, and differentiation rinse back blue. Slices were dehydrated, transparent, and sealed. The staining results were observed and interpreted under a light microscope. The positive part of cell is the cytoplasm, which is yellowish-brown.

### 2.4. Statistics

We performed statistical analyses using the SPSS 21.0 statistical software (SPSS, Chicago, IL). Correlations of tumor budding, cell nest size, and TBNS system with clinicopathologic parameters were calculated using the *χ*2 and Fisher's exact test. Survival analyses were performed using the Kaplan–Meier and log-rank test. Multivariate survival analyses were performed using Cox proportional-hazards model. A *p* value ≤ 0.05 was considered significant.

## 3. Results

### 3.1. Study Sample: General Features

Patients' median age was 66 years (range 41 to 85 years); 56 were male, and 31 were female. 23 cases were stage I, 31 cases were stage II, 22 cases were stage III, and 11 cases were stage IV. The mean follow-up time for patients was 55 months (11 to 119 months). 38 (43.7%) patients died during follow-up, and 23 (26.4%) patients were disease-specific death. The detailed clinicopathologic parameters are shown in Table 1.

### 3.2. Study Sample: Histomorphologic Features

Of 87 samples, 12 cases were low-grade urothelial carcinoma, whereas 75 cases were high-grade urothelial carcinoma. Budding activity was absent in 60 tumors (68.9%), 19 (21.8%) showed low budding activity, and 8 (9.3%) showed high budding activity. The smallest invasive tumor cluster within the entire tumor area (small cell nest size) was large sized in 32 cases (36.8%), medium sized in 17 cases (19.5%), and small sized in 30 cases (34.5%) and was single-cell invasion in 8 cases (9.2%). The TBNS grade combining of tumor budding and cell nest size scores was G1 (well differentiated) in 48, G2 (moderately differentiated) in 30, and G3 (poorly differentiated) in 8 cases (Table 1).

### 3.3. Correlation of Tumor Budding, the Cell Nest Size, and the TBNS Grade with Clinicopathologic Features

Tumor budding activity positively correlated to lymphovascular invasion, peripheral nerve invasion, pT, and tumor stage (*p* = 0.025, *p* = 0.042, *p* < 0.001, and *p* = 0.001, respectively). The cell nest size positively correlated with pT and tumor stage (*p* < 0.001 and *p* < 0.001, respectively). Neither tumor budding nor tumor cell size correlated with age, sex, side, tumor size, number, and WHO grade. The TBNS grading system was closely related to peripheral nerve invasion, WHO grade, pT, and tumor stage (*p* = 0.045, *p* = 0.037, *p* < 0.001, and *p* < 0.001, respectively) not to other clinicopathologic features (Table 1).

The article "A Novel Prognostic Stratified System Based on Tumor Budding and the Cell Nest Size in Ureter Urothelial Carcinoma" was retracted in 2023. Reasons: signs of a paper mill; suspected computer-generated content; unreliable results or conclusions; concerns about the data.

### 3.4. Correlation of Tumor Budding, the Cell Nest Size, and the TBNS Grade with Survival

Tumor budding activity significantly correlated to OS, DFS, and DSS (*p* < 0.001). The mean DSS was 62.6 months in patients with no budding activity in their tumors, 46.4 months when their tumors had low budding activity, and 25.9 months when their tumors had high budding activity (Table 1 and Figure 2).

The l cell nest size significantly correlated to OS, DFS, and DSS (*p* < 0.01). The mean DSS was 69.1 months in patients with a large nest size, 60.8 months in patients with a medium nest size, 45.0 months in patients with a small nest size, and 31.4 months in patients with single-cell invasions (Table 1 and Figure 3).

The TBNS grading system significantly correlated with OS, DFS, and DSS (*p* < 0.001) (Figure 4). The mean DSS was 66.2 months in well-differentiated tumors (G1, score 2–3), 46.5 months in moderately differentiated tumors (G2, score 4–5), and 25.9 months in poorly differentiated tumors (G3, score 6–7).

Multivariate survival analyses showed that the TBNS grading system was an independent prognostic factor for DFS and DSS (*p* = 0.007 and *p* = 0.045, respectively). Relative to G1, the DFS hazard ratio for G2 tumors was 0.547 (95% confidence interval: 0.041–7.284) and 10.492 (95% confidence interval: 2.296–47.948) for G3 tumors. Relative to G1, the DSS hazard ratio for G2 tumors was 0.939 (95% confidence interval: 0.059–14.946) and 11.498 (95% confidence interval: 1.500–88.117) for G3 tumors (Table 2).

## 4. Discussion

Ureter carcinoma is a rare malignant tumor of the upper urinary tract, which seriously threatens human health. Its morbidity and mortality are increasing year by year [2]. The clinical staging of ureter carcinoma is determined based on the depth of tumor invasion, lymph node metastasis, and distant metastasis. Therefore, cancer staging is beneficial to the evaluation of disease prognosis and the selection of treatment plan [3]. However, due to the heterogeneity of individual tumors, patients with ureteral cancer within the same tumor stage have different outcomes. Therefore, it is necessary to combine some new morphological and molecular markers into pTNM staging to stratify patients' prognostic risk more reasonably and accurately.

The article "A Novel Prognostic Stratified System Based on Tumor Budding and the Cell Nest Size in Ureter Urothelial Carcinoma" was retracted in 2023. Reasons: signs of a paper mill; suspected computer-generated content; unreliable results or conclusions; concerns about the data.

Increasing studies have confirmed that tumor budding is a risk factor for highly invasive and poor prognosis of malignant tumors. Rogers et al. meta-analysis showed that tumor budding is a strong adverse prognostic factor for cancer recurrence, 5-year cancer-related mortality, and lymph node metastasis in colorectal cancer and proposed that its inclusion in CRC staging facilitates effective risk stratification for colorectal cancer [25].

Tumor budding has rarely been studied in upper urinary tract urothelial carcinoma (UUTUC). Kawamura et al. investigated 135 invasive UUTUCs, in which high tumor budding correlated to the pT stage, lymphovascular invasion, and lymph node metastasis, and confirmed that tumor budding is associated with poor prognosis of UUTUCs [26]. The cell nest size especially a smaller cell nest size is the second histological feature that predicts clinical biological behavior of tumor aggressiveness. Tumor budding and cell nest size have similar morphological features, which can be observed in the same tumor and associated with invasive biological behavior; these characteristics indicate that tumor budding and cell nest size may have internal relations.

Recently, new grading systems based on tumor budding and cell nest size (TBNS grade system) have been introduced for use in squamous cell carcinoma of different anatomical regions including the lung [20], oral cavity [22], larynx and hypopharynx [23], esophagus [21], and uterine cervix. Zare et al. [19] evaluated the association of tumor budding, cell nest size, and other morphologic factors with clinical pathological parameters in 157 cases of larynx and hypopharynx squamous cell carcinoma. The results confirmed that the three-tiered novel grade system based on tumor budding and the cell nest size is the highly independent prognostic factor of squamous cell carcinoma of the larynx and hypopharynx and obviously better than the current WHO staging scheme. Boxberg et al. [23] selected 94 cases of cervical squamous cell carcinoma with no neoadjuvant therapy, pT1b or higher stage, and continuous surgical resection, and scored the tumor budding and cell nest size. The results showed that the higher grade of tumors in the TBNS system was closely associated with the advanced pathological stage and lymph node metastasis. The authors suggested that the TBNS grading system has excellent prognostic performance and applicability in the stratification of cervical squamous cell carcinoma [19]. This novel grading system was initially applicable for squamous cell carcinoma in resected specimens, but Jesinghaus et al. investigated its usefulness in pretherapeutic biopsy specimens. They named this grading system as the cellular dissociation grade, which could stratify prognosis and predict the infiltrative depth and lymphatic metastasis [27]. Recently, the applicability of the TBNS grading system in malignancies other than squamous cell carcinoma has been discussed. Shi et al. explored the application of this novel grading system in 398 cases with surgical resection, no neoadjuvant therapy, and higher than the pT1a stage in endocervical adenocarcinoma. The three-tiered grading system was closely related to shorter overall survival and tumor recurrence. Furthermore, the overall survival of HPV-associated adenocarcinoma and gastric-type adenocarcinoma could be stratified via this grading system [24]. However, this novel TBNS grading system has not been investigated in ureter urothelial carcinoma yet.

The article "A Novel Prognostic Stratified System Based on Tumor Budding and the Cell Nest Size in Ureter Urothelial Carcinoma" was retracted in 2023. Reasons: signs of a paper mill; suspected computer-generated content; unreliable results or conclusions; concerns about the data.

In this study, we explored the prognostic significance of the TBNS grading system based on tumor budding and the cell nest size in 87 surgically resected ureter urothelial carcinoma. Confirming the results previously generated for squamous cell carcinoma and adenocarcinoma, TBNS grade was strongly related to peripheral nerve invasion, WHO grade, pT, tumor stage, and shorter survival (OS, DSS, and DFS). It was also an independent prognostic factor for DSS and DFS in ureter urothelial carcinoma. The results showed that the tumor stage was an independent prognostic factor for OS and DSS; therefore, the tumor stage and TBNS grading system could satisfactorily predict DSS of ureteral urothelial carcinoma and the TBNS grade had an advantage in predicting DFS of this cancer. These findings suggested that the TBNS grading system was a histopathologic-based prognostic indicator and might influence clinical decision-making.

Our study had some limitations. Firstly, our results are based on a small cohort and our study is a single-center study and they should be verified using a larger cohort to explore the utility of the TBNS system in daily pathologic diagnosis. Secondly, we did not include lymph nodes in our study. Lymphadenectomy was performed in China during a few urinary tract surgeries. In radical nephroureterectomy, lymph node dissection is disputed. Due to the lower incidence and few prospective studies, current evidence supports lymphadenectomy for accurate tumor staging [28]; however, there is a disagreement regarding its effect on improving prognosis. Its specific indications and scope needed more prospective randomized controlled trials.

The article "A Novel Prognostic Stratified System Based on Tumor Budding and the Cell Nest Size in Ureter Urothelial Carcinoma" was retracted in 2023. Reasons: signs of a paper mill; suspected computer-generated content; unreliable results or conclusions; concerns about the data.

In conclusion, the novel TBNS system based on tumor budding and the cell nest size is an ideal prognostic indicator in resected uterine urothelial carcinoma. It still needs to be further explored its role in biopsy and neoadjuvant therapy specimens of this cancer type.

## Figures and Tables

**Figure 1:** Morphologic features of ureter urothelial carcinoma (HE). (a, b) Tumor budding: (a) low budding and (b) high budding; (c) cell nest size: single-cell invasion; (d) CK immunohistochemical staining. Arrows represent tumor budding.

**Figure 2:** Association of the tumor budding with overall survival (a), disease-specific survival (b), and disease-free survival (c), in ureter urothelial carcinoma.

**Figure 3:** Association of the cell nest size with overall survival (a), disease-specific survival (b), and disease-free survival (c), in ureter urothelial carcinoma.

**Figure 4:** Association of the TBNS grade with overall survival (a), disease-specific survival (b), and disease-free survival (c), in ureter urothelial carcinoma.

**Table 1:** Correlation of tumor budding, cell nest size, and TBNS system with clinicopathological parameters in ureter urothelial carcinoma.

	Tumor budding *p*				Cell nest size *p*					TBNS grade *p*			
	Without	Low	High		>15 cells	5–15 cells	2–4 cells	Single cell		G1	G2	G3	
	60	19	8		32	17	30	8		49	30	8	
Age				0.584					0.888				0.731
≤median	33	9	3		17	9	16	3		26	16	3	
>median	27	10	5		15	8	14	5		23	14	5	
Sex				0.677					0.973				0.797
Male	37	14	5		20	11	19	6		30	20	6	
Female	23	5	3		12	6	11	2		19	10	2	
Side				1.000					0.593				0.300
Left	33	11	4		15	9	19	5		24	20	4	
Right	27	8	4		17	8	11	3		25	10	4	
Size				0.498					0.556				0.946
≤median	38	9	5		18	12	16	6		30	17	5	
>median	22	10	3		14	5	14	2		19	13	3	
Number				1.000					0.544				0.515
Single	50	16	7		26	13	26	8		39	27	7	
Multiple	10	3	1		6	4	4	0		10	3	1	
WHO grade				0.052					0.053				**0.037**
Low	12	0	0		8	3	1	0		11	1	0	
High	48	19	8		24	14	29	8		38	29	8	
LVI				**0.025**					0.139				0.058
0	47	11	3		24	14	20	3		38	20	3	
1	13	8	5		8	3	10	5		11	10	5	
PNI				**0.042**					0.078				**0.045**
0	47	12	3		25	15	18	4		39	20	3	
1	13	7	5		7	2	12	4		10	10	5	
pT				**<0.001**					**<0.001**				**<0.001**
1	21	2	0		14	7	2	0		21	2	0	
2	23	7	3		12	7	10	4		19	11	3	
3	16	10	1		6	3	17	1		9	17	1	
4	0	0	4		0	0	1	3		0	0	4	
Stage				**0.001**					**<0.001**				**<0.001**
I	21	2	0		14	7	2	0		21	2	0	
II	21	7	3		12	6	9	4		18	10	3	
III	14	8	0		5	4	13	0		9	13	0	
IV	4	2	5		1	0	6	4		1	5	5	

**Table 2:** Multivariate analysis for overall survival, disease-specific survival, and disease-free survival in ureter urothelial carcinoma.

	OS		DSS		DFS	
	HR (95% CI)	*p*	HR (95% CI)	*p*	HR (95% CI)	*p*
*Age*	3.669 (1.631-8.254)	**0.002**	—	—	—	—
*LVI*	2.340 (0.943-5.805)	0.067	3.298 (1.099-9.893)	**0.033**	1.215 (0.547-2.696)	0.633
*PNI*	1.461 (0.610-3.502)	0.395	1.017 (0.363-2.847)	0.975	4.851 (2.130-11.047)	**<0.001**
*Tumor budding* ^a,b^		0.467		0.179		0.900
Tumor budding (1)	1.632 (0.436-6.101)	0.467	3.508 (0.562-21.900)	0.179	1.070 (0.371-3.085)	0.900
*Cell nest size* ^a,b^		0.598		0.527		0.310
Cell nest size (1)	0.965 (0.294-3.165)	0.953	0.342 (0.032-3.678)	0.376	0.515 (0.105-2.516)	0.412
Cell nest size (2)	0.438 (0.088-2.169)	0.312	0.485 (0.059-3.977)	0.500	4.763 (0.458-.49.487)	0.191
*TBNS grade*		0.238		**0.045**		**0.007**
TBNS grade (1)	2.925 (0.565-15.314)	0.201	0.939 (0.059-14.946)	0.964	0.547 (0.041-7.284)	0.648
TBNS grade(2)	3.810 (0.637-22.797)	0.14**3**	11.498 (1.500-88.117)	0.019	10.492 (2.296-47.948)	**0.00**2
*pT* ^a,b^		**0.004**		**0.002**		0.149
pT (1)	7.891 (0.523-118.971)	0.136	88.641 (4.107-1913.212)	**0.004**	19.818 (0.986-398.287)	0.051
pT (2)	0.301 (0.032-2.811)	0.292	0.899 (0.069-11.680)	0.935	3.447 (0.467-25.459)	0.225
*Stage*		**<0.001**		**<0.001**		0.099
Stage (1)	0.074 (0.003-1.919)	0.117	0.014 (0.000-0.994)	0.050	0.043 (0.001-1.344)	0.073
Stage (2)	3.136 (0.229-42.902)	0.392	4.147 (0.139-123.700)	0.412	0.558 (0.049-6.406)	0.640
Stage (3)	27.904 (1.850-420.920)	0.016	158.695 (3.904-6450.986)	0.007	1.014 (0.087-11.819)	0.991

^a^Reduction of degrees of freedom due to constants or linearly dependent covariates. ^b^Constant or linearly dependent covariable pT; (3): stage (1) + stage (2) + stage (3)-pT (1)-pT (2); cell nest size (3) = TBNS grade (1) + TBNS grade (2)-cell nest size (2); tumor budding (2) = TBNS grade (2).

The article "A Novel Prognostic Stratified System Based on Tumor Budding and the Cell Nest Size in Ureter Urothelial Carcinoma" was retracted in 2023. Reasons: signs of a paper mill; suspected computer-generated content; unreliable results or conclusions; concerns about the data.

## Data Availability

All analyses of the data have been reported in the Supporting Information File. In case any other clarification is needed, the relevant information will be made available with permission from the corresponding author.
